# A Novel Missense Mutation of Arginine Vasopressin Receptor 2 in a Chinese Family with Congenital Nephrogenic Diabetes Insipidus: X-Chromosome Inactivation in Female CNDI Patients with Heterozygote 814A>G Mutation

This article has been retracted.

**DOI:** 10.1155/2022/7073158

**Published:** 2022-07-12

**Authors:** Li Zang, Yuping Gong, Yijun Li, Jingtao Dou, Zhaohui Lyu, Xiaoqing Su, Yawei Zhang, Yiming Mu

**Affiliations:** ^1^Department of Endocrinology, The First Medical Center of Chinese PLA General Hospital, Beijing 100853, China; ^2^Department of Endocrinology, Jiangxi Pingxiang People's Hospital, Pingxiang 337055, China

## Abstract

**Background:**

To identify novel clinical phenotypic signatures of congenital nephrogenic diabetes insipidus (CNDI).

**Methods:**

A Chinese family with CNDI was recruited for participation in this study. The proband and one of his uncles suffered from polydipsia and polyuria since infancy. The results of clinical testing indicated the diagnosis of CNDI. 10 family members had similar symptoms but did not seek medical advice. Genetic testing of mutations in the coding region of the aquaporin 2 (*AQP2*) gene and the arginine vasopressin receptor 2 (*AVPR2*) gene were carried out in 11 family members. Somatic DNA from 5 female family members was used to test for methylation of polymorphic CAG repeats in the human androgen receptor (AR) gene, as an index for X-chromosome inactivation pattern (XCIP).

**Results:**

*AQP2* gene mutations were not found in any family members, but a novel missense mutation (814th base A>G) in exon 2 of the *AVPR2* gene was identified in 10 individuals. This mutation leads to a Met 272 Val (GAT-GGT) amino acid substitution. Skewed X-chromosome inactivation patterns of the normal X allele were observed in 4 females with the *AVPR2* gene mutation and symptoms of diabetes insipidus, but not in an asymptomatic female with the *AVPR2* gene mutation.

**Conclusions:**

Met 272 Val mutation of the *AVPR2* gene was identified as a novel genetic risk factor for CDNI. The clinical NDI phenotype of female carriers with heterozygous *AVPR2* mutation may be caused by X-chromosome inactivation induced by dominant methylation of the normal allele of *AVPR2* gene.

## 1. Introduction

Congenital nephrogenic diabetes insipidus (CNDI) is a relatively rare genetic disorder which is characterized by renal resistance to the antidiuretic effects of arginine vasopressin (AVP), an antidiuretic hormone (ADH) that is produced in the posterior pituitary and functions as a regulator of the kidney's ability to reabsorb water. 90% of cases with CNDI are caused by mutations of arginine vasopressin type 2 receptor (*AVPR2*) gene, which encodes the vasopressin V2 receptor [1]. The remaining 10% of cases with CNDI are caused by mutations of aquaporin-2 (*AQP2*), a water channel gene located on chromosome 12q13. In particular, mutations of *AQP2* are linked to autosomal recessive or dominant forms of CNDI [2]. The *AVPR2* gene is located on the long arm of the X-chromosome (Xq28), and mutations of *AVPR2* gene can cause CNDI in an X-linked recessive manner. To date, approximately 250 *AVPR2* mutations have been identified and the inheritance pattern is often used to distinguish various forms of CNDI [3]. Most of the female carriers with *AVPR2* mutations are asymptomatic. However, some female carriers with *AVPR2* mutations may experience symptoms of polydipsia and polyuria, due to their impaired ability to concentrate urine, as is observed in male patients with skewed X-chromosome inactivation.

In this study, we identify novel clinical phenotypic signatures of CNDI through genetic analysis of mutations in *AQP2* and *AVPR2* in a Chinese family with autosomal CNDI, which was confirmed by both clinical examination and the mode of inheritance. We found a novel mutation of the *AVPR2* gene, and this newly identified *AVPR2* mutation is considered the potential pathogeny of CNDI, because skewed X-chromosome inactivation was confirmed as the reason for symptoms in the female patients carrying this mutation.

## 2. Materials and Methods

This study was approved by the ethics committee of our institutions. Written informed consent was obtained from all participants in this study. The investigation was performed in adherence with the ethical principles of the Helsinki Declaration.

### 2.1. Analysis of Clinical Data

The pedigree of the Chinese family described in this study is presented in Figure 1. The proband (subject III-6) was a 31-year-old male, who was admitted to our department because of polydipsia, polyuria, and nocturia since infancy. His 24-hour urine volume was 5-6 L/24 h. The results of his urinary laboratory examination indicated marked hypernatremia (s-Na 155 mmol/L) along with hypoosmotic polyuria (urinometry 1.002-1.004). Serum urine nitrogen (9.6 mmol/L) and serum creatinine (140.2 *μ*mol/L) were mildly elevated. Pituitary magnetic resonance imaging (MRI) showed visible bright spots in the posterior pituitary. The pituitary was normal in appearance, without evidence of a hypothalamic mass (Figure 2). Computed tomography (CT) of the urinary system revealed bilateral ureterectasis and hydronephrosis combined with right kidney atrophy (Figure 2). Tests of the capacity for water deprivation and vasopressin loading revealed that dehydration and subcutaneous injection of 5 units of vasopressin did not increase the concentration of urine osmolality (Table 1). These findings supported the diagnosis of CNDI. The symptoms of polydipsia and polyuria were relieved, and the 24 h urine volume was controlled at 2000 mL after he was treated with hydrochlorothiazide and indomethacin. One of his uncles (subject II-2) suffered from the same symptoms, including bilateral ureterectasis and hydronephrosis. Measurements of urine osmolality obtained during water deprivation and vasopressin loading tests showed that the patient had lost the renal response to the injection of vasopressin. Hydrochlorothiazide treatment was proved effective. The other members of this pedigree, including his grandmother (subject I-1), another uncle (subject II-6), his mother and three aunts (subjects II-3, 4, 5, and 7), his brother and two cousins (subjects III-5, 3, and 4), and his 2-year-old nephew (subject IV-1), had developed varying degrees of diabetes insipidus, but they did not seek medical advice.

### 2.2. Genomic DNA Extraction and Sequence Analysis

11 members of the family (including subjects II-1, 2, 3, 4, and 6; III-3, 4, 5, 6, and 7; and IV-1) provided written consent after being informed of the study's purpose. Five milliliters of peripheral blood samples was collected and placed into a tube with ethylenediaminetetraacetic acid (EDTA). Genomic DNA was extracted using a kit (Qiagen, Duesseldorf, Germany). To amplify the *AVPR2* and *AQP2* genes, polymerase chain reaction (PCR) was performed using primers for *AVPR2* and *AQP2* genes as previously reported [4, 5]. After the purification of PCR products, automated DNA-sequencing was performed using an instrument (310 Genetic Analyzer; ABI Prism) and the BigDye kit (Applied Biosystems, USA).

### 2.3. X-Chromosome Inactivation Pattern Analysis

Among methylation sites on the inactive X-chromosome, the first exon of the human androgen receptor (AR) gene is typically used to analyze the X-chromosome inactivation pattern by counting the polymorphic CAG repeats in exon 1 of the AR gene [6]. Genomic DNA samples obtained from 5 female members (subjects II-3 and 4; III-3 and 4 with symptoms of diabetes insipidus; and subject III-7 without symptoms) were pretreated with bisulfite for DNA methylation detection using the EpiTect Bisulfite Kit (Qiagen) according to the manufacturer's instructions. Briefly, genomic DNA samples were digested by two methylation-sensitive restriction enzymes (HpaII and HhaI). Restriction enzyme (RE) digestion was designed to yield cleavage only at RE sites on the active X-chromosome, but not on the inactive methylated X-chromosomes. Then, RE-digested DNA samples were used for PCR amplification of the AR locus, including the HpaII and HhaI cleavage sites and the CAG repeat element. The primers for this study were designed as previously reported [7]. After 4% agarose gel electrophoresis, two bands of the PCR products were detected: 280 bp from one allele and 292 bp from another allele. The density of each band was quantified by scanning with Band scan software. The degree of X-chromosome inactivation for each allele was expressed as a percentage of the inactive X-chromosome. The value or percentage of relative X-chromosome inactivation for one allele was determined by calculations using the following equation: N280/(N280 + N292) × 100. The pattern of X-chromosome inactivation was considered to be skewed if the percentage of X-chromosome inactivation was ≥80%. Values ranging from 50% to 80% were considered to indicate a random pattern of X-chromosome inactivation.

## 3. Results

### 3.1. Mutations of the AVPR2 and AQP2 Genes

Genomic DNA sequencing was performed for the precise diagnosis of CNDI using the samples obtained from 11 family members. Because of the initial suggested diagnosis of autosomal CNDI, the sequence of the entire coding region of the *AQP2* gene in each DNA sample was examined, but no variation was found in any of the family members recruited for this study. In the proband, two hemizygous mutations (814th base A>G and 927th base A>G) were found in the 2nd and 3rd exons of the *AVPR2* gene, respectively (Figures 3(a) and 3(c)). The A>G mutation in the 927th base of the 3rd exon suggested a silent Leu 309 Leu (TAG-TAC) mutation, while the A>G mutation at the 814th base of the 2nd exon resulted in an amino acid substitution (Met 272 Val, i.e., from GAT to GGT) in the *AVPR2*. A hemizygous Met 272 Val mutation was also found in some male family members with symptoms of diabetes insipidus, such as subjects II-2 and 6; III-5; and IV-1. Heterozygous Met 272 Val mutations were found in some female family members with symptoms of diabetes insipidus (subject II-3 and 4 and III-3 and 4) (Figures 3(b) and 3(d)), as well as one asymptomatic female member (subject III-7). No *AVPR2* gene mutation was detected in one asymptomatic male family member (subject II-1). The Met 272 Val mutation was considered responsible for the morbidity associated with CNDI, and it was not found in the 100 unrelated healthy individuals used as controls.

### 3.2. Assay for X-Chromosome Inactivation

Both 280-bp and 292-bp PCR products of the AR locus were examined for the analysis of X-chromosome inactivation. Digestion of the DNA samples with two methylation-sensitive REs prior to PCR resulted in a difference in density between the bands. Our study found that the percentages of relative X-chromosome inactivation for one allele were 90%, 83%, 87%, 85%, and 39% in subjects II-3 and 4, III-3 and 4, and subject III-7, respectively (Table 2). These findings indicated nonrandom X-chromosome inactivation in subjects II-3 and 4 and III-3 and 4 but not in subject III-7. We explored the relationship between the age of the female subjects and the percentage of relative X-chromosome inactivation, and no correlation between two variables was found.

## 4. Discussion

In this study, 12 members of a Chinese family suffered from polydipsia and polyuria from infancy were diagnosed with CNDI. An autosomal CNDI pedigree was considered because male as well as female members of the family were affected. Surprisingly, no mutations in the coding region of the *AQP2* gene, which was linked to autosomal recessive or dominant forms of CNDI, were detected in any of the family members, while genetic analysis of *AVPR2* gene revealed a novel mutation of 814th base A>G, which induced Met 272 Val amino acid substitution. The 814th base A>G mutation had not been reported previously and was suggested responsible for CNDI. The CNDI in this pedigree was considered to be an X-linked recessive inherited disease, with involvement in female patients caused by skewed inactivation of the X-chromosome.

CNDI was first described by McIlraith in 1892. Patients with CNDI mainly present with persistent polyuria, polyuria, dehydration, delayed growth, and intellectual disability. Laboratory examinations usually reveal hypernatremia and hyposthenuria that do not respond to exogenous AVP [2]. Because of persistent polyuria and delays in diagnosis, many of the patients have dysfunction of the kidney, such as urinary retention, hydroureter, hydronephrosis, and mild renal insufficiency. In this study, the 31-year-old proband and one of his uncles were diagnosed with CNDI based on their presentation of clinical symptoms, results of laboratory examinations, and positive response to hydrochlorothiazide and indomethacin. Numerous other family members (males and females) also had symptoms of diabetes insipidus. So this pedigree was first considered as evidence of autosomal dominant CNDI caused by the *AQP2* gene mutation. However, no variation in *AQP2* was found in any family members.

Further analysis revealed two hemizygous mutations in the exons of *AVPR2* in the proband, which indicated a diagnosis of X-linked recessive inherited disease in this family. van den Ouweland first reported that mutation of the *AVPR2* gene was linked to X-linked recessive CNDI in 1992 [8]. Moreover, 50% of *AVPR2* gene mutations are missense mutations [9]. There are three types of *AVPR2* gene mutations, which are differentiated based on the function and subcellular localization of mutant proteins [10]. In Type 1, the mutant receptors are located on the cell surface, with impaired ligand binding, leading decreased cAMP production. In Type 2, the mutant receptors are not transported to the cell surface, accumulating instead in a pre-Golgi compartment, due to defective intracellular transport. In Type 3, the mutant receptors are expressed at low levels because of the rapid degradation of unstable mRNA. The 927A>G *AVPR2* mutation harbored by the proband is a nonsense mutation reported in the literature as the most common polymorphism of this gene [11]. However, the 814A>G mutation found in our study is a novel missense mutation that causes a Met 272 Val substitution. In this family, hemizygous mutation of Met 272 Val was also found in some male family members with symptoms of diabetes insipidus, while heterozygous mutations of Met 272 Val were found only in female family members (with or without symptoms). However, the Met 272 Val mutation was not found in asymptomatic male members. These results suggested that the novel mutation identified in this study was responsible for V2 receptor dysfunction. The Met 272 Val mutation occurred in a transmembrane region of the V2 receptor, which may lead to improper assembly of the V2 receptor. Another study identified a different mutation (Met 272 Lys) at this residue in a patient with CNDI, resulting in insertion of a charged residue in the transmembrane domain, causing a failure to signal upon stimulation with AVP [12]. Other studies identified an *AVPR2* gene mutation at a residue next to position Thr273Met in Turkish and Spanish patients. The Thr273Met mutation is also located in the region that codes for the transmembrane domain, which affects proper assembly and function of the V2 receptor [13, 14]. The amino acid residue at positions 272 and 273 is vital for the structure of the V2 receptor, and the Met 272 Val mutation was not found in 100 unrelated healthy individuals used as controls. Therefore, based on previous reports, the novel mutation found in our study could be classified as a Type 1 mutation that was pathognomonic for CNDI. Further basic research is needed to investigate the potential effects of the 814A>G mutation on V2 receptor function.

In our study, there were 4 female patients with CNDI and *AVPR2* mutations. Female CNDI patients with the *AVPR2* mutations are usually diagnosed as a carrier of heterozygous mutation and asymptomatic. Therefore, it is necessary to test for other gene mutations related to CNDI for female patients, especially those affecting the *AQP2* gene, which have an autosomal dominant pattern of transmission. In our study, direct sequence analysis did not reveal any mutations in *AQP2* among all tested family members. *AQP2* mutations were not pathognomonic for CNDI among female members of this pedigree. The reason why female carriers of mutation of *AVPR2* gene showed NDI symptoms would be explain by skewed X-inactivation. As we know, X-chromosome inactivation occurs early in female embryogenesis at about the 32-to-64 cell stage, when there are few progenitor cells for a given tissue. X-chromosome inactivation is irreversible and affects all descendants of a given progenitor cell. Skewed inactivation of the X-chromosome bearing the normal AVPR2 allele may suppress the expression of AVPR2 protein with normal function, leading to female carriers with an NDI phenotype. In this study, we examined CAG repeat polymorphisms at the AR locus in DNA samples to measure X-chromosome inactivation in female carriers. Female members of the pedigree with *AVPR2* mutation and symptoms of diabetes insipidus displayed X-chromosome inactivation, while this phenomenon did not appear in asymptomatic female members with *AVPR2* mutation, indicating that X-chromosome inactivation was responsible for the symptoms observed in female patients. There were 5 pedigrees with skewed X-inactivation in female carriers of *AVPR2* mutation had been reported [15–19]. Nomura et al. first reported 3 male members diagnosed with CNDI with *AVPR2* mutation (a G inserted at nucleotide 804 of the open reading frame). Three female individuals in the pedigree displayed different degrees of symptoms of NDI, and all of them possessed both the normal and abnormal genes. The X-inactivation patterns of the female members were investigated via the detection of methylated trinucleotide repeat in the human AR gene. The grandmother showed extremely skewed methylation of one X-chromosome, and the mother revealed moderately skewed methylation. The daughter of the grandmother's sister, who had no symptoms of NDI, showed random methylation. The highly skewed X-inactivation pattern of the grandmother suggested that her NDI phenotype was caused by dominant methylation of the normal allele of V2R gene [15]. Kinoshita et al. reported a pedigree of CNDI with a Japanese female proband (two-nucleotide deletion change at codon 30 (g.452-453delAC) in the V2R gene, resulting in a frameshift and premature termination in translation at codon 190). The X-chromosome inactivation pattern detection using methylation analysis of the polymorphic CAG repeat in the AR gene revealed that the value for relative X-chromosome inactivation of one allele was 70.2% [16]. Satoh et al. reported the value for relative X-chromosome inactivation was 71.6%-93% in female carriers with AVPR2 mutation who showed clinical symptoms, while it was only 60.7%-61.9% in asymptomatic female carriers [17–19]. The results of our study are consistent with other previous observations of females with X-linked NDI. In previous reports, the ratios of X-chromosome inactivation for a given tissue were similar among individuals, but in a normal female, those ratios may vary depending on cell lineage [20]. Presumably, the X-chromosome inactivation pattern in leucocytes from blood samples may not precisely reflect that in renal tubular cells. Owing to difficulty in obtaining renal tubular tissue for this study, further research is needed to explore X-chromosome inactivation in the kidneys of females with NDI.

## 5. Conclusions

In conclusion, a novel *AVPR2* mutation (814A>G) in a Chinese family with CNDI has been identified in this study. This novel mutation may be involved in improper assembly of the V2 receptor. Female carriers with the heterozygous form of the 814A>G mutation had a clinical NDI phenotype, perhaps due to the pattern of X-chromosome inactivation. The clinical NDI phenotype in female carriers with the heterozygote 814A>G mutation may result from the methylation coded for by the normal allele of the *AVPR2* gene, which is dominant. It is necessary to perform functional studies in the future to investigate the effects of the Met272Val mutation on the V2 receptor on terms of intracellular localization, ligand binding, and adenylate cyclase activation.

## Figures and Tables

**Figure 1:** The pedigree of the Chinese family with congenital nephrogenic diabetes insipidus. Solid symbols denote the affected individuals. The arrow indicates the proband.

**Figure 2:** The imaging feature of the proband. (a) Pituitary MRI showed normal anterior and posterior pituitary. (b) Urinary system CT scan showed bilateral ureterectasis and hydronephrosis combined with right kidney atrophy.

**Figure 3:** Sequence analysis of the 2nd and 3rd exons in AVPR2 gene. (a, b) sequencing in the 814th base of 2nd exon, A was substitute of G which resulted a Met 272 Val (GAT-GGT) amino acid substitution. A was hemizygous mutation in the male subjects, B was heterozygous mutation in the female subjects. (c, d) sequencing in the 927th base of 3rd exon, A was substitute of G which suggested a silent mutation Leu 309 Leu. C was hemizygous mutation in the male subjects; D was heterozygous mutation in the female subjects.

**Table 1:** Results on the water deprivation and vasopressin test of proband.

Time (hours)	Urine volume (mL)	Urine specific gravity	Plasma osmolality (mOsm/L)	Body weight (kg)
1	150	1.002	307.1	51
2	190	1.003	306.9	51
3	150	1.003	312.2	51
4	100	1.002	305.5	50.5
5	70	1.002	306.9	51
6∗	60	1.003	311.6	51
7	80	1.002	311.2	50.8

Note: 5U vasopressin was subcutaneously injected at the beginning of the 6th hour.

**Table 2:** Analysis of the X-chromosome inactivation pattern in the family.

	Subjects				
	II-3	II-4	III-3	III-4	III -7
Fragment length allele 1 (bp)	280	280	280	280	280
Fragment length allele 2 (bp)	292	292	292	292	292
Percentage of cells with allele 1 as inactive X-chromosome (%)	90	83	87	85	39
Percentage of cells with allele 2 as inactive X-chromosome (%)	10	17	13	15	61

## Data Availability

The datasets generated during and/or analyzed during the current study are not publicly available but are available from the corresponding author on reasonable request. The sequencing data were deposited in the ClinVar database (http://www.ncbi.nlm.nih.gov/clinvar; accession number: SCV001469055).

## Abbreviations

CNDI: Congenital nephrogenic diabetes insipidus
AVP: Arginine vasopressin
ADH: Antidiuretic hormone
*AVPR2*: Vasopressin type 2 receptor
*AQP2*: Aquaporin-2
PCR: Polymerase chain reaction.

## References

[1] Yoo T. H., Ryu D. R., Song Y. S. (2006). Congenital nephrogenic diabetes insipidus presented with bilateral hydronephrosis: genetic analysis of V2R gene mutations. *Yonsei Medical Journal*.

[2] Morello J. P., Bichet D. G. (2001). Nephrogenic diabetes insipidus. *Annual Review of Physiology*.

[3] Bockenhauer D., Bichet D. G. (2017). Nephrogenic diabetes insipidus. *Current Opinion in Pediatrics*.

[4] Çelebi Tayfur A., Karaduman T., Özcan Türkmen M. (2018). A novel mutation in the *AVPR*2 gene causing congenital nephrogenic diabetes insipidus. *Journal of Clinical Research in Pediatric Endocrinology*.

[5] Rugpolmuang R., Deeb A., Hassan Y., Deekajorndech T., Shotelersuk V., Sahakitrungruang T. (2014). Novel AQP2 mutation causing congenital nephrogenic diabetes insipidus: challenges in management during infancy. *Journal of Pediatric Endocrinology & Metabolism*.

[6] Lexner M. O., Bardow A., Juncker I. (2008). X-linked hypohidrotic ectodermal dysplasia. Genetic and dental findings in 67 Danish patients from 19 families. *Clinical Genetics*.

[7] Allen R. C., Zoghbi H. Y., Moseley A. B., Rosenblatt H. M., Belmont J. W. (1992). Methylation of HpaII and HhaI sites near the polymorphic CAG repeat in the human androgen-receptor gene correlates with X chromosome inactivation. *American Journal of Human Genetics*.

[8] van den Ouweland A. M., Dreesen J. C., Verdijk M. (1992). Mutations in the vasopressin type 2 receptor gene (*AVPR*2) associated with nephrogenic diabetes insipidus. *Nature Genetics*.

[9] Böselt I., Tramma D., Kalamitsou S. (2012). Functional characterization of novel loss-of-function mutations in the vasopressin type 2 receptor gene causing nephrogenic diabetes insipidus. *Nephrology, Dialysis, Transplantation*.

[10] Fujiwara T. M., Bichet D. G. (2005). Molecular biology of hereditary diabetes insipidus. *Journal of the American Society of Nephrology*.

[11] Shen Y., Lai X., Xiao X. (2014). Genetic analysis of a congenital nephrogenic diabetes insipidus pedigree. *Chinese Medical Journal*.

[12] Wildin R. S., Cogdell D. E., Valadez V. (1998). AVPR2 variants and V2 vasopressin receptor function in nephrogenic diabetes insipidus. *Kidney International*.

[13] Duzenli D., Saglar E., Deniz F., Azal O., Erdem B., Mergen H. (2012). Mutations in the AVPR2, AVP-NPII, and AQP2 genes in Turkish patients with diabetes insipidus. *Endocrine*.

[14] García Castaño A., Pérez de Nanclares G., Madariaga L. (2015). Novel mutations associated with nephrogenic diabetes insipidus. A clinical-genetic study. *European Journal of Pediatrics*.

[15] Nomura Y., Onigata K., Nagashima T. (1997). Detection of skewed X-inactivation in two female carriers of vasopressin type 2 receptor gene mutation. *The Journal of Clinical Endocrinology and Metabolism*.

[16] Kinoshita K., Miura Y., Nagasaki H., Murase T., Bando Y., Oiso Y. (2004). A novel deletion mutation in the arginine vasopressin receptor 2 gene and skewed X chromosome inactivation in a female patient with congenital nephrogenic diabetes insipidus. *Journal of Endocrinological Investigation*.

[17] Satoh M., Ogikubo S., Yoshizawa-Ogasawara A. (2008). Correlation between clinical phenotypes and X-inactivation patterns in six female carriers with heterozygote vasopressin type 2 receptor gene mutations. *Endocrine Journal*.

[18] Faerch M., Corydon T. J., Rittig S., Christensen J. H., Hertz J. M., Jendle J. (2010). Skewed X-chromosome inactivation causing diagnostic misinterpretation in congenital nephrogenic diabetes insipidus. *Scandinavian Journal of Urology and Nephrology*.

[19] Morin D. (2014). Vasopressin V2 receptor-related pathologies: congenital nephrogenic diabetes insipidus and nephrogenic syndrome of inappropiate antidiuresis. *Néphrologie & Thérapeutique*.

[20] Sharp A., Robinson D., Jacobs P. (2000). Age- and tissue-specific variation of X chromosome inactivation ratios in normal women. *Human Genetics*.

